This article has been retracted.

# Mechanical Characteristics and Permeability Characteristics of Dry-Hot Rock Mass

**DOI:** 10.1155/2023/5298404

**Published:** 2023-07-07

**Authors:** Dong Yang, Changsong Lu, Wuqing Wen, Hanlie Cheng, David Cadasse

**Affiliations:** ^1^Downhole Services Company, CNPC Bohai Drilling Engineering Company Limited, Renqiu 062552, Hebei, China; ^2^School of Energy Resource, China University of Geosciences, Beijing 434000, China; ^3^COSL-EXPRO Testing Services (Tianjin) Co. Ltd., Tianjin 300457, China; ^4^The King's School, BP1560, Bujumbura, Burundi

## Abstract

As a rock mass with shallow burial, high temperature, and large-scale development, the study of its mechanical and seepage characteristics plays an important role in the efficient development of geothermal energy. With the development of geothermal energy in China, a breakthrough has been made in the exploration of dry-hot rocks, and the realization of efficient development of dry-hot rocks has become the focus of attention. Systematic research on rock mechanics and seepage characteristics of dry-hot rocks has become a key research topic. Granite is the most typical dry-hot rock. In this paper, granite in the Qinghai area is selected as the research object, and experiments on physical characteristics, mechanical parameters, and seepage characteristics of granite are carried out to study the effects of different depths and temperatures on mechanical parameters and seepage characteristics of granite. The results show that the physical parameters of granite in Qinghai do not change obviously with the increase of depth, and granite has the characteristics of low water absorption and low porosity. At the same time, the parameters of water absorption and porosity at different depths are close, and the dispersion is small, so the rocks are very dense. The rocks have relatively high P-wave velocity and low S-wave velocity, and the elastic wave velocity changes little at different depths. With the increase of confining pressure, the strength of granite rock increases. Under different confining pressures, the rock shows brittle failure characteristics after the peak stress. According to Hoek–Brown and Mohr–Coulomb strength curves, the strength value is 173.52 MPa. After high temperature treatment, a complex fracture network is formed in the granite. With the increase of temperature, the permeability and porosity of the granite increase continuously, and 500°C is the temperature threshold. When the temperature is lower than 300°C and the stress is less than 30 MPa, the granite has negative Poisson's ratio, and the permeability and effective stress of dry-hot rocks are piecewise linear functions. The research results provide theoretical guidance for fracturing of dry-hot rocks and exploitation of geothermal energy.

## 1. Introduction

With the rapid development of economy, energy shortage has become an important factor hindering the development of global economy. As a new energy source, geothermal energy is clean, safe, and easy to exploit [1]. Geothermal energy development and utilization rose in 1950s. With the rapid growth of energy demand, geothermal energy exploitation entered a period of rapid development [2]. As geothermal energy storage rock mass, dry-hot rock has great potential and development prospect and has become an irreplaceable important energy source in China's sustainable development [3].

Granite, as the most important dry-hot rock, has the characteristics of shallow burial, high temperature, and exploitable utilization. At present, the research on granite mainly focuses on genesis, resource evaluation, exploration methods, etc., while the research on mechanics and seepage characteristics of dry-hot rocks is less [4, 5]. Some researchers have carried out triaxial loading and unloading experiments and microstructure analysis of granite. With the increase of confining pressure, Poisson's ratio and elastic modulus of granite also increase [6]. The mechanical properties and anisotropy of fine-grained granite are studied. The confining pressure has an influence on the failure mode of fine-grained granite. Under the condition of low confining pressure, the fine-grained granite breaks and forms a complex fracture network [7, 8]. Some researchers have carried out triaxial compression on granite in different areas. Under low confining pressure, the granite is mainly cracked and double shear, while under high confining pressure, the granite is mainly single shear [9]. Some researchers have studied the characteristics of permeability, deformation, and anisotropy of granite with the change of confining pressure and analyzed the microstructure of samples by SEM, revealing the reasons of permeability and deformation of granite [10]. Some researchers have developed instruments to measure the physical characteristics and porosity of low-permeability rocks and have used this instrument to carry out low-permeability and porosity experiments on granite core samples [11]. Some researchers have carried out triaxial seepage experiments of granite under different axial pressures, confining pressures, and air pressures and analyzed the influence of stress and gas slippage effect on the permeability k_0_ of granite [12]. It is found that k_0_ is negatively exponentially related to stress difference and stress gradient at a lower pressure gradient, and the attenuation is most significant when the pressure gradient is 0∼0.2 MPa. According to the nanoscale pore characteristics of granite, some researchers have analyzed the seepage characteristics of granite under different stress conditions [13–15]. The results show that the flow produced by Darcy flow is directly proportional to pressure, pressure gradient, and permeability.

As a rock mass with shallow burial, high temperature, and large-scale development, the study of its mechanical and seepage characteristics plays an important role in the efficient development of geothermal energy [16–18]. Systematic study of the mechanical and seepage characteristics of dry-hot rock mass has become a key research topic. Granite is the most typical dry-hot rock. In this paper, the granite in the Qinghai area is taken as the research object, and the physical, mechanical, and seepage characteristics of granite with different depths are studied experimentally [19–21]. The effects of different depths and temperatures on the mechanical and seepage characteristics of granite are studied, which provides theoretical guidance for the fracturing of dry-hot rock and the exploitation of geothermal energy [22].

## 2. Sample Preparation and Test Methods

### 2.1. Sample Preparation

The core is taken from the outcrop of Indosinian granite in Qinghai area, and it is medium-fine grained and porphyritic, mainly composed of Shi Ying, feldspar, and biotite. In this paper, granite cores at different drilling depths (100 m, 200 m, 300 m, 400 m, 500 m, and 600 m) are selected (Figure 1), which are mainly medium-fine porphyritic granodiorite. See Table 1 for information of core collection. After the core obtained by drilling is marked, it is kept in good condition by the sampling box, which reduces the damage caused by strong disturbance during transportation.

The diameter of the drilled core obtained onsite is 63 mm, and the rock samples meeting the test standards are prepared through fine processing by rock coring machine, cutting machine, and grinding machine. According to GB/T 50266-99 and SL264-2001, when rock is subjected to triaxial compression test, the specimen should be a cylinder with a diameter of 48 mm∼54 mm, a height-diameter ratio of 2.0∼2.5, an allowable deviation of height and diameter of ±0.3 mm, and unevenness of both ends of the specimen. In this paper, the processing size of the core is required to be Φ50 × 100 m, as shown in Figure 2.

### 2.2. Test Plan and Test Method

#### 2.2.1. Testing of Petrophysical Parameters

Before obtaining the mechanical characteristics of rock, it is necessary to count the physical parameters of rock samples. In this paper, the block density, particle density, water content, water absorption, porosity and wave velocity parameters of drill cores at different depths are tested. Four rock samples are selected for each depth, totaling 24, and the average values of the samples at different depths are counted as the physical parameters of rock testing. Measure the diameter, length, and quality of the test by using vernier caliper and electronic scale. The direct wave is used to measure the longitudinal wave velocity of the sample. The specific steps are as follows: the wave transducers are placed at the axial ends of the sample and clamped, and the transducers and the sample are coupled with vaseline. The instrument records data every 0.1 *μ*s to calculate the longitudinal wave velocity of the sample.  Table 2 shows the basic physical parameters of samples with different depths.

#### 2.2.2. Rock Mechanics Test

Rock mechanical parameters include uniaxial and triaxial compressive strength, tensile strength, and shear strength. The domestic standard of engineering rock mass test method and the suggested method of rock mechanics test put forward by the International Society of Rock Mechanics is adopted for the experiment. Triaxial compression test was carried out on granite rock samples according to relevant specifications.

The triaxial compression test of rock mass in this paper is completed by the MTS815.03 pressure test system (Figure 3). The press is produced by MTS Company of the United States, which mainly carries out conventional mechanical tests of rock, concrete, and other materials, and is equipped with a servo-controlled fully automatic triaxial compression and measurement system. The system consists of loading part, testing part, control part, and program control. The maximum vertical pressure of the system is 4600 kN, the maximum vertical deformation is 100 m, the maximum confining pressure is 140Mpa, and the overall stiffness of the test frame is 11.0 × 109 N/m.

The MTS rock mechanics test system is used to carry out triaxial compression test of rock, and the deformation parameters and triaxial strength parameters of rock under different confining pressures are obtained. The test process is as follows:

1. The heat-shrinkable tube is sleeved on the core, heated and shrunk by a hot air gun, and the core is fixed between the upper and lower pressure heads. The heat-shrinkable tube can fix the core well and isolate the core from direct contact with silicone oil.
2. After the heat-shrinkable tube is heated, the core will be heated to cause radial shrinkage. To prevent the measurement error caused by heating, the heated core should stand at room temperature for more than 5 h.
3. Install the radial strain sensor in the middle of the core, put it into the triaxial chamber, lower the confining cylinder, lock the bolt tightly, inject hydraulic oil (dimethyl silicone oil), and exhaust the gas.
4. After the confining pressure cylinder is filled, add confining pressure to the triaxial chamber, and load it to the predetermined confining pressure value at a rate of about 5 MPa per minute, and load the confining pressure to the specified value at a rate of 2 MPa/min.
5. Start the axial loader, adopt axial strain control, and carry out axial loading at the rate of 0.02%/min. When the sample is suddenly destroyed, the system will automatically stop, and there is a good back zone of stress-strain relationship. When the load is close to zero, the test will be stopped manually.

After the completion of the test, the damaged samples were treated with Nano Vox EL-3502E micro-CT observation heat treatment to analyze the spatial distribution of cracks. The experimental steps are as follows: the sample is fixed on the gripper, and the crosscut gray image of the sample is obtained by scanning it in CT scanning room. The fracture distribution of the core was obtained by 3D reconstruction.

#### 2.2.3. Rock Seepage Test

Granite has the characteristics of small porosity and low permeability, and the permeability directly affects the heat extraction of granite. In this paper, the pulse attenuation test method is used to test the permeability change law of granite. In this experiment, HPPD-100 pulse attenuation permeameter produced by GCTS Company of the United States was used, and the effective permeability range was 10 nd–1 md. Before the pulse penetration test, first fully saturate the pore fluid in the sample. Main test steps are as follows:

1. Fill the system pipeline and container with fluid and apply a small pressure from the pore pressure booster
2. Open a part of the valves, let the pore liquid flow out, open the feedback channel of the displacement sensor of the pore pressure booster, push the liquid with the booster, and let the liquid flow out from the upper pressure head
3. Adopting a pore pressure supercharger to push the liquid, flowing out of the lower pressure head, installing the saturated sample, and sealing with a heat-shrinkable tube
4. Close the pressure chamber, apply a small contact load and confining pressure, and achieve the preloading state; use the pore pressure booster to apply appropriate pressure and wait for a few minutes, and then close the valve
5. Clear the differential pressure sensor, slowly discharge the lower pressure until the read data reaches the preset pressure difference, and check the readings of the two pressure sensors until the balance point is reached

During the test, the pore pressure should be kept at 1 MPa and the differential pressure should be 250 KPa. By pressurizing with water purification, the deviating stress of confining pressure is always kept at about 1 MPa, and the permeability is measured once every 3 MPa increase and once every 10 MPa when the effective stress is greater than 20 MPa.

## 3. Experimental Results and Analysis

### 3.1. Physical Experiment Results of the Sample

Physical parameters of rock samples were obtained by physical tests. As can be seen from Table 1, the water content of granite rock samples is 0.08%–0.09%, the saturated water absorption is 0.33%–0.35%, the total porosity is 0.84%–0.87%, and the P-wave velocity is above 3300 m/s. The granodiorite is characterized by high density, low water content, low water absorption, and low porosity. The rock is very dense, with good mineral cementation and uniform grain development.

### 3.2. Mechanical Test Results of Samples

Triaxial compression tests of granite samples under 5 MPa, 10 MPa, 15 MPa, and 20 MPa are carried out in this test.  Figure 4 shows the stress-strain relationship in the process of loading failure of the samples under different confining pressures. It can be seen from Figure 4 that, during the loading process of the sample, the first stage is compaction, but this stage is not obvious because of the dense granite. After the sample enters the elastic stage, the stress and strain are linearly positively correlated until the sample reaches the peak strength. After the peak strength of the sample, there is no ductility behavior, but it falls linearly directly and finally reaches the residual strength. At the same time, with the increase of confining pressure, the yield stage becomes obvious, and the ductility stage gradually becomes obvious after the peak strength. The damaged rock and rock mass still have high residual strength, which can be loaded again.

Triaxial compression test results (Table 3) of samples with a depth of about 100 m under different confining pressures are selected. From the table, it can be seen that the peak strength of the rock increases with the increase of confining pressure, and the axial deformation of the rock reaches 0.63 mm when it reaches the peak strength. With the increase of confining pressure, the residual strength also increases, and the strength is still above 80 MPa.

According to the experimental results, the deformation and strength of the sample change obviously with the increase of confining pressure. Because the contact degree between mineral grains is randomly distributed, the deformation effect of each mineral component is different, which leads to the change of the internal stress field. Under the action of stress, the microcracks of the sample close, and the strength is determined by the friction of grains. Therefore, the friction between grains in the shear plane is high, so the residual strength is high.

The denaturation characteristics of rock are mainly represented by Young's modulus and peak strain. Young's modulus mainly includes elastic modulus and deformation modulus. The elastic modulus refers to the slope of the approximate straight line part of the axial stress-axial strain curve of the sample, and the deformation modulus refers to the slope of the line connecting the sample with the origin at 50% axial stress.  Figure 5 shows the variation diagram of Young's modulus of rock samples with confining pressure. From the fitting curve in the figure, it can be seen that, with the increase of confining pressure, Young's modulus of rock samples increases and the sensitivity of deformation modulus and elastic modulus of rock samples to confining pressure is basically the same. This is mainly due to the strong connection force and close contact between granite mineral particles, which causes little deformation in the initial compression stage and is not obvious in the compaction stage.

With the increase of confining pressure, the triaxial compressive strength of the specimen increases. Under different confining pressures, granite samples show brittle failure characteristics after peak stress. According to the triaxial compression strength data of the samples, the Hoek–Brown and Mohr–Coulomb strength curves and strength parameter values of granite samples are calculated (Figure 6). It can be seen from the figure that the strength of granite is 173.52 MPa, the internal friction angle *φ* is 56.79, and the cohesion C is 29.27 MPa.

### 3.3. Experimental Results of Sample Seepage

According to the sample seepage experiment, the permeability of the sample under different effective stress is counted, as shown in Table 4. It can be seen from Table 4 that the permeability of the sample decreases gradually with the increase of effective stress: when the effective stress is less than 21 MPa, the permeability of the sample decreases rapidly with the increase of effective stress. When the effective stress exceeds 21 MPa, with the increase of stress, the permeability of the sample still decreases, but the decreasing range obviously decreases. At the same time, it is found that there is a piecewise linear function between the permeability and effective stress of granite, which is mainly due to the negative Poisson's ratio of granite. When the confining pressure and effective stress of granite increase, the negative Poisson's ratio of granite leads to the increase of its radial shrinkage. When compressed to a certain extent, the negative Poisson's ratio of dry-hot rock is suppressed, and the decrease of permeability decreases. When the confining pressure is 0 MPa, the negative Poisson's ratio of the sample is the most obvious. With the increase of confining pressure, the radial shrinkage of the sample gradually decreases. When the confining pressure exceeds 30 MPa, the negative Poisson's ratio phenomenon gradually disappears.

According to the CT scanning image, the internal structure of granite is very dense, and there are no obvious holes or cracks. However, after high-temperature heating, a large number of cracks are produced in the rock and connected with each other, forming a complex crack network. When the granite is treated at 500°C, the cracks will extend horizontally and vertically, forming a grid-like crack network. With the increase of temperature, the porosity and permeability of the sample increase obviously. When the temperature reaches 500°C, the increase is the largest, and the porosity increases from 3.6% to 7.0%. The permeability increases from 0.08 md to 0.82 md, which increases by an order of magnitude. Therefore, it can be considered that, about 500°C is the threshold temperature for the change of granite physical properties. When the hot dry rock is lower than this threshold temperature, the heat is affected by adsorbed water and interlayer water. When the temperature is higher than the threshold, a large number of new pores are generated in the rock mass and connected with each other, and the permeability increases rapidly.

According to the statistics of the accumulated heat production at different injection velocities, it can be seen that the heat production gradually increases with the increase of the flow velocity. When the flow velocity exceeds 42 kg/s, the total heat production reaches the peak value of 5.8 × 1013 J. After that, the total heat production begins to decrease with the increase of the flow velocity, which is mainly affected by the negative Poisson's ratio. During geothermal exploitation, by injecting cold water into the rock reservoir for heat exchange, the temperature of dry hot rock around the production well gradually decreases. The injected water pressure causes the pore pressure to increase and the effective stress of rock to decrease gradually. When the temperature drop of the rock mass exceeds a certain value, the phenomenon of negative Poisson's ratio begins to appear in the dry hot rock, which greatly affects the permeability of the fracture and reduces the heat recovery rate. Therefore, in the actual geothermal development, the injection speed of cold water needs to be controlled reasonably, and the greater the injection speed, the worse the effect will actually be. Increasing the injection velocity can obviously improve the heat recovery rate, but it will shorten the life of the whole heat recovery system and may also lead to the decline of the final heat recovery. In the actual production, the water injection speed should be controlled reasonably to ensure the heat production efficiency and avoid the negative Poisson's ratio effect of dry-hot rock as much as possible.

## 4. Conclusion

Dry-hot rock is a kind of rock mass with shallow burial, high temperature, and large-scale development. With the large-scale development of geothermal energy in China, the exploration of dry-hot rocks has become a key concern, and systematic research on rock mechanics and seepage characteristics of dry-hot rocks has become a key research topic. Granite is the most typical dry-hot rock. Taking granite in Qinghai as the research object, this paper studies the mechanical parameters and seepage characteristics of granite with different depths and temperatures and obtains the mechanical properties and seepage characteristics of dry-hot rock, which provides theoretical guidance for the fracturing of dry-hot rock and exploitation of geothermal energy. The main research results are as follows:

1. Through physical test, the water content of granite samples is 0.08% ∼ 0.09%, the saturated water absorption is 0.33% ∼ 0.35%, the total porosity is 0.84% ∼ 0.87%, and the longitudinal wave velocities are all above 3,300 m/s. Triaxial compression tests were carried out on granite samples under different confining pressures. With the increase of confining pressures, the peak strength of granite samples increased and was above 200 MPa. At the same time, when the rock reached the peak strength, the axial deformation reached 0.63 mm, and the residual strength also increased and was above 80 MPa. With the increase of confining pressure, Young's modulus of the sample increases. The experimental statistics show that the strength of granite is 173.52 MPa, the internal friction angle *φ* is 56.79, and the cohesion C is 29.27 MPa.
2. The internal structure of granite is very dense, with no obvious holes or cracks. After high temperature heating, a large number of cracks are produced in the rock and connected with each other, forming a complex crack network. Through seepage experiment, the permeability of the sample decreases gradually with the increase of effective stress. At the same time, when the effective stress is less than 21 MPa, the permeability of the sample decreases rapidly with the increase of effective stress. When the effective stress exceeds 21 MPa, the permeability of the sample still decreases with the increase of stress, but the decrease is obviously reduced. At the same time, it is found that there is a piecewise linear function between the permeability and effective stress of granite, which is mainly due to the negative Poisson's ratio of granite. When compressed to a certain extent, the negative Poisson's ratio of dry-hot rock is suppressed, and the decrease of permeability decreases. When the confining pressure is 0 MPa, the negative Poisson's ratio of the sample is the most obvious. With the increase of confining pressure, the radial shrinkage of the sample gradually decreases. When the confining pressure exceeds 30 MPa, the negative Poisson's ratio phenomenon gradually disappears. In the process of water injection for heat recovery, the effect will be worse if the water injection rate is too fast. When the water injection rate is greater than a certain value, the accumulated heat recovery is smaller than that at low flow rate. In this paper, the mechanical and seepage characteristics of dry-hot rock are studied, and the experimental results obtained have strong regularity, which has certain reference significance for the geothermal development of dry-hot rock.

## Figures and Tables

**Figure 1:** Granite core.

**Figure 2:** Rock sample diagram.

**Figure 3:** MTS rock mechanics test system.

**Figure 4:** Stress-strain relationship during loading failure of specimens under different confining pressures.

**Figure 5:** Changes of Young's modulus-confining pressure of the sample.

**Figure 6:** Strength curve of granodiorite (490m∼510 m) in borehole TH01.

**Table 1:** Core collection records.

Serial number	Sample number	Sampling point		Sample length (m)	Sample name
		Huiji	Start-end (m)		
1	QH01	83 (1/3)	93.41∼93.08	67	Medium-fine porphyritic biotite granodiorite
2	QH01	157 (4/5)	201.33∼201.45	12	
3	QH01	227 (5/7)	301.98∼304.32	34	
4	QH01	283 (1/1)	400.82∼402.25	43	
5	QH01	330 (2/6)	501.89∼503.55	66	
6	QH01	372 (5/6)	599.33∼603.09	76	

**Table 2:** Basic physical parameters of samples with different depths.

Drilling depth (m)	Average diameter (mm)	Average height (mm)	Average mass (g)	Moisture content (%)	Saturated water absorption (%)	Total porosity (%)	Longitudinal wave velocity (ms^−1^)
100	50.04	100.41	467.1	0.091	0.342	0.851	3535.56
200	50.42	99.98	468.49	0.089	0.345	0.843	3447.33
300	50.58	99.91	471.97	0.092	0.341	0.847	3362.63
400	50.37	100.23	480.49	0.091	0.345	0.862	3457.84
500	50.41	100.13	482.09	0.087	0.337	0.856	3653.88
600	50.94	99.94	463.9	0.088	0.338	0.860	3460.75

**Table 3:** Triaxial compression test results of samples under different confining pressures.

Core number	Confining pressure (MPa)	Modulus of elasticity (GPa)	Poisson's ratio	Triaxial compressive strength (MPa)
1	5	51.07	0.233	233.13
2	10	51.27	0.24	302.16
3	15	51.25	0.30	378.68
4	20	52.07	0.29	418.29

**Table 4:** Changes of permeability of specimen with effective stress.

Effective stress (MPa)	1	3	6	9	12	15	18	21	30	40	50	60
Sample permeability (md)	0.90	0.89	0.75	0.63	0.46	0.44	0.43	0.35	0.31	0.26	0.21	0.18

## Data Availability

The figures and tables used to support the findings of this study are included in the article.
